# The role of phosphatidylserine recognition receptors in multiple biological functions

**DOI:** 10.1186/s11658-020-00214-z

**Published:** 2020-03-26

**Authors:** Mehri Bemani Naeini, Vanessa Bianconi, Matteo Pirro, Amirhossein Sahebkar

**Affiliations:** 1 Nanotechnology Research Center, Pharmaceutical Technology Institute, Mashhad University of Medical Sciences, Mashhad, Iran; 2 Unit of Internal Medicine, Angiology and Arteriosclerosis Diseases, Department of Medicine, University of Perugia, Perugia, Italy; 3 Halal Research Center of IRI, FDA, Tehran, Iran; 4 Neurogenic Inflammation Research Center, Mashhad University of Medical Sciences, Mashhad, Iran; 5 Department of Medical Biotechnology, School of Medicine, Biotechnology Research Center, Pharmaceutical Technology Institute, Mashhad University of Medical Sciences, P.O. Box: 91779-48564, Mashhad, Iran

**Keywords:** Apoptosis, Efferocytosis, Macrophage, Phosphatidylserine, Phosphatidylethanolamine, Receptor

## Abstract

Apoptotic cells are rapidly engulfed and degraded by phagocytes through efferocytosis. Efferocytosis is a highly regulated process. It is triggered upon the activation of caspase-dependent apoptosis, which in turn promotes the expression of “eat me” signals on the surface of dying cells and the release of soluble “find me” signals for the recruitment of phagocytes. To date, many “eat me” signals have been recognized, including phosphatidylserine (PS), intercellular adhesion molecule-3, carbohydrates (e.g., amino sugars, mannose) and calreticulin. Among them, PS is the most studied one. PS recognition receptors are different functionally active receptors expressed by phagocytes. Various PS recognition receptors with different structure, cell type expression, and ability to bind to PS have been recognized. Although PS recognition receptors do not fall into a single classification or family of proteins due to their structural differences, they all share the common ability to activate downstream signaling pathways leading to the production of anti-inflammatory mediators. In this review, available evidence regarding molecular mechanisms underlying PS recognition receptor-regulated clearance of apoptotic cells is discussed. In addition, some efferocytosis-independent biological functions of PS recognition receptors are reviewed.

**This article was specially invited by the editors and represents work by leading researchers.**

## Introduction

Efferocytosis is the clearance of apoptotic cells by either professional phagocytes, including macrophages and dendritic cells (DCs), or non-professional phagocytes, that is neighboring tissue cells (e.g., endothelial cells, epithelial cells, fibroblasts) acquiring a phagocyte-like phenotype [1–3]. At the earliest steps of cell death, soluble “find-me” signals attract phagocytes towards dying cells [4–7]. Subsequently, the exposure of phosphatidylserine (PS) on the apoptotic cell surface has a crucial role in facilitating specific recognition of dying cells by phagocytes [8] and triggering phagocytic cup formation [9]. PS, a negatively charged phospholipid normally confined to the inner plasma membrane leaflet by flippases, is externalized on the apoptotic cell surface by scramblases [6, 10–12]. Several molecules, including secreted soluble proteins [e.g., growth arrest-specific gene 6 (Gas6), protein S (ProS), and milk-fat globule epidermal growth factor 8 (MFG-E8)] and type I membrane proteins expressed on the phagocyte surface (e.g., CD300) may recognize PS. Ligation between PS on the apoptotic cell surface and PS recognition receptors is essential for phagocyte cup formation and engulfment [13]. In fact, the inhibition of either PS or PS recognition receptors has been reported to be sufficient to block apoptotic cell removal by phagocytes [14, 15]. Noteworthy, other molecules apart from PS have been recognized as “eat me” signals on the apoptotic cell surface [e.g., intercellular adhesion molecule-3 (ICAM-3), carbohydrates, and calreticulin] [16–20] (Fig. 1). However, whether their ligation with specific phagocyte receptors may further augment engulfment remains to be clarified [21]. In addition, a phospholipid other than PS [i.e., phosphatidylethanolamine (PE)] is asymmetrically expressed on the surface of apoptotic cells. However, its specific role in apoptosis has not been fully clarified. In this review, we will discuss the role of PS recognition receptors in efferocytosis. In addition, some efferocytosis-independent biological functions of PS recognition receptors will be reviewed.

**Fig. 1:** Recognition of apoptotic cells by phagocytes. Numerous receptors on the phagocyte membrane interact with “eat me” signals on the apoptotic cell surface either directly or indirectly through bridging molecules. Apoptotic cells can attract phagocytes through the release of soluble molecules, namely “find me” signals. Instead, healthy cells express “don’t eat me” molecules to avoid phagocytosis. BAI1, brain-specific angiogenesis inhibitor-1; C1q, complement component 1q; FcR, Fc fragment of immunoglobulin G receptor; Gas6, growth arrest-specific gene 6; ICAM-3, intracellular adhesion molecule-3; LOX-1, lectin-like oxidized low-density lipoprotein receptor-1; LRP, LDL receptor-related protein; PS, phosphatidylserine; MerTK, c-mer proto-oncogene tyrosine kinase; MFG-E8, milk-fat globule epidermal growth factor 8; PSR, PS receptor; SRA, scavenger receptor class A; TIM-4, transmembrane immunoglobulin and mucin domain protein 4; αVβ3, vitronectin receptor; β2GPI, beta 2-glycoprotein 2

### Exposure of PS: apoptotic and non-apoptotic role

Generally, exposure of PS on the membrane of apoptotic cells leads to cell removal by phagocytes through efferocytosis. In physiological conditions, as efferocytosis occurs efficiently and swiftly, it is hard to find free apoptotic corpses throughout body tissues, even when large numbers of cells undergo apoptosis. Such effective clearance of cells that are no longer desired or are functionally abnormal is crucial for the maintenance of tissue homeostasis and for the prevention of various diseases including cancer [22, 23], degenerative diseases of the central nervous system, atherosclerosis and autoimmune diseases [24–28]. Therefore, efferocytosis mediators may represent potential therapeutic targets for either the prevention or the treatment of these pathological conditions [29–31].

However, the binding between PS and the PS recognition receptor has a regulatory role also in different efferocytosis-independent biological processes [e.g., platelet activation [32], osteoblast-mediated mineralization [33], cell fusion [34], viral infections [35]]. Reportedly, PS exposure has a crucial role in axonal fusion, that is, the process in which a regrowing axon reconnects with its detached segment, leading to the structural and functional restoration of the injured neuron [36]. PS externalization, by facilitating cell-cell contact between myoblasts, seems to play a regulatory role in the early phases of myotube formation, that is, the fusion of an individual myoblast into multinucleated cells differentiating into myocytes [34]. PS is externalized by trophoblasts and mediates intertrophoblastic fusion during placental development [37]. Non-apoptotic macrophages are known to externalize PS and recognition of PS-expressing macrophages by CD36 triggers macrophage fusion, thereby mediating the formation of multinucleated giant cells [38, 39].

Moreover, PS exposure has a crucial role in different infections. The presence of PS on the surface of some enveloped and non-enveloped viruses (i.e., apoptotic mimicry) has been reported to promote viral infectivity by facilitating viral entry in host cells expressing PS recognition receptors and enhancing immune escape by infected cells [40–42]. In addition, during infections by different pathogens [e.g., human immunodeficiency virus (HIV), hepatitis C virus (HCV), *Plasmodium*, *Leishmania* or *Mycobacterium leprae*], anti-phospholipid antibodies, including anti-PS, are detectable in the serum of a high percentage of patients [43, 44]. In the case of *Plasmodium* infection, the binding between anti-PS antibodies and infected PS-exposing erythrocytes has been suggested to have a crucial role in the removal of intracellular pathogens. Indeed, although infected PS-exposing erythrocytes express high levels of CD47, a “do-not-eat-me” signal [45], their interaction with anti-PS antibodies mediates their phagocytosis and exerts a protective effect against *Plasmodium* [44]. Furthermore, the binding of soluble PS released by tumor cells to the PS receptor (PSR) has been shown to result in the production of anti-inflammatory mediators that block antitumor immune responses [e.g., tumor growth factor (TGF)-β, interleukin (IL)-10 and prostaglandin E2 (PGE2)] [46].

Several members of the galectin family induce the exposure of PS on the surface of inflammatory cells. However, Gal-1- and Gal-3-induced externalization of PS promote differential responses in T cells and neutrophils. Gal-3, but not Gal-1, induces both PS exposure and apoptosis in primary activated human T cells, whereas both Gal-1 and Gal-3 induce PS exposure but not cell death in neutrophils. Noteworthy, although in some conditions galectin-induced PS exposure does not occur in cells undergoing apoptosis, it can induce cell paraparesis, that is, sensitization to phagocytic clearance [47]. Indeed, in some circumstances galectin-induced PS exposure is independent of evident alterations in mitochondrial potential, caspase activation, membrane morphology or cell death typically seen in apoptotic cells [47]. Also, it may be fully reverted after galectin removal without determining any subsequent alteration in cell viability [47]. Such phagocytic removal of living cells promoted by Gal-1 and Gal-3-induced PS externalization represents a peculiar model of cellular turnover and regulation of various cellular processes, including cellular trafficking and immunological synapse formation [48, 49].

### PS recognition receptors

#### Biological functions of PS recognition by TAM family members/ProS/Gas6

Axl (also known as UFO),Tyro3 and Mer are members of a subfamily of receptor tyrosine kinases (RTKs) named TAM (from the first letters of Tyro3, Axl, and Mer) [50]. They were identified as PS recognition receptors by using anti-PS antibodies to screen the human cDNA expression library from B lymphoblastoid λgt11 [51], and by polymerase chain reaction (PCR) amplification using degenerate oligonucleotides [52]. Axl, Tyro3 and Mer bind to the carboxy terminal domains of their ligands (i.e., ProS and Gas6) [53], which in turn bind to PS through their amino terminal domains [54–56], thereby acting as ‘bridges’ between PS on apoptotic cells and TAM receptors on phagocytes [57]. Noteworthy, ProS has no affinity for Axl [58], while Gas6 binding to Axl occurs with a higher affinity as compared to Gas binding to Mer and Tyro3 [59]. Upon ligation with either ProS or Gas6, the dimerization of TAM receptors occurs, leading to the phosphorylation of tyrosine residues in their cytoplasmic region [60] and to the activation of different downstream signaling pathways.

TAM receptors may be variably expressed in different tissues and cell types. Tyro3 is expressed in prostate, cerebral cortex and olfactory bulb. Axl is expressed in lipopolysaccharide-treated macrophages, osteoblasts, uterus and ovary. Mer is expressed in resident peritoneal macrophages, lung, small intestine and retinal pigment epithelial cells [13].

Under physiological conditions, TAM receptors are involved in either efferocytosis-dependent or efferocytosis-independent biological processes, including the regulation of inflammatory cytokine release, cell proliferation/survival, cell adhesion and migration, platelet activation and thrombus formation [61, 62].

Several studies have recognized the oncogenic role of the abnormal expression of TAM receptors in a wide variety of tumors [63, 64]. One the one hand, excessive TAM receptor activation may promote tumor immune escape through the induction of an immunosuppressive response in the tumor microenvironment [65–67]. On the other hand, TAM receptor activation may stimulate tumor cell proliferation and survival by increasing the production and release of TGF-β [68]. Therefore, therapeutic inhibition of TAM receptors may represent a potential strategy to inhibit tumor progression [69, 70].

Moreover, TAM receptors have been reported to have a crucial role in the regulation of immune response in different pathological conditions. Accordingly, the inhibition of TAM receptor-activated intracellular signaling pathways has been suggested to have a therapeutic role in the treatment of sepsis and post-transplantation organ rejection [71]. By contrast, sustained TAM receptor inhibition has been associated with the pathogenesis of various autoimmune diseases, including systemic lupus erythematosus and rheumatoid arthritis [66, 72–74].

Finally, a variable association has been described between TAM receptor activation and atherosclerosis progression. Accordingly, defective Mer function has been reported to induce the accumulation of apoptotic foam cells and the formation of necrotic cores within atherosclerotic plaques [75–77], whereas Gas6 binding to TAM receptors has been shown to promote atherogenesis by increasing endothelial activation, monocyte chemotaxis and vascular smooth muscle cell (VSMC) differentiation into foam cells [78, 79].

#### Biological functions of PS recognition by TIM family members

Members of the transmembrane immunoglobulin and mucin domain (TIM) family are a group of proteins (i.e., TIM-1, TIM-2. TIM-3, TIM-4) which are variably expressed on the inflammatory cell surface and have a crucial role in the regulation of immune responses. The TIM family consists of three members in humans and four members in mice [80]. Among them, TIM-1 and TIM-4 act as PS recognition receptors, whereas TIM-2 and TIM-3 do not have noticeable PS-binding activity [81].

TIM-1, also known as kidney injury molecule-1 (KIM-1), is a type 1 membrane receptor [82]. It is a proximal tubular cell (PTC) surface protein which is expressed in a wide range of kidney diseases. Upon PS recognition [83] it mediates the conversion of tubular epithelial cells into non-professional phagocytes [84], thereby promoting efferocytosis of apoptotic cells and exerting a protective effect against acute kidney injury [85–90]. However, KIM-1 binding to PS exerts nephroprotective action also through efferocytosis-independent mechanisms, that is, the limitation of renal epithelial cell damage through the inhibition of Gα12 [91] or the promotion of tubular epithelium repair through activation of the extracellular signal-regulated kinase (ERK)/mitogen-activated protein (MAP) kinase (MAPK) signaling pathway [92].

Moreover, KIM-1 also plays an immunoregulatory role by controlling Th2, Th1, and Th17 cell differentiation [93] and the activation of B cells, DCs, and natural killer (NK) cells [94]. Specifically, KIM-1-mediated efferocytosis induces a pro-tolerogenic immune response, leading to the inhibition of CD4 T-cell proliferation and to the activation of regulatory T cells [95].

TIM-4 is expressed in a variety of resident macrophages, including peritoneal macrophages, hepatic Kupffer cells, skin CD169+ macrophages [59, 96] and CD4+ tangible body macrophages at Peyer patches of the small intestine [97]. It binds to PS via the IgG domain. TIM-4 itself is not able to mediate efferocytosis [98] and requires TAM receptors [59]. Accordingly, macrophages expressing both TIM-4 and TAM receptors (e.g., skin macrophages, resident peritoneal macrophages and Kupffer cells) [59] engulf apoptotic cells in two steps, that is, tethering and tickling [99]. In the tethering step, TIM-4 firmly binds to PS and recruits apoptotic cells to the macrophage surface. In the tickling step, soluble “bridge” proteins (e.g., ProS, Gas6 and MFG-E8) bind to PS on the apoptotic cell surface and to PS recognition receptors on phagocytes, thereby promoting phagocytic cup formation and engulfment. In different tumors TIM-4 has been described as an oncogenic driver which promotes tumor cell proliferation and facilitates immune escape by tumor cells through the induction of an immunosuppressive response in the tumor microenvironment [100–102].

#### Biological functions of other PS recognition receptors

Many other cell surface molecules have been shown to recognize PS, including brain-specific angiogenesis inhibitor 1 (BAI1), lectin-like oxidized low-density lipoprotein receptor-1 (LOX-1), stabilin-1 and stabilin-2, CD300a, CD300b, CD300f, receptor for advanced glycosylation end products (RAGE), complement component 1q (C1q), β2-glycoprotein I (β2GPI), annexins, integrins αVβ3/β5, and PSR [103]. Some of these PS recognition receptors have signaling ability, while others mainly act as tethering and adhesion molecules. Their role in multiple biological functions will be discussed in the following section.

#### Biological functions of PS recognition by annexins, β2GPI and C1q

All annexin family molecules, except for one, act as bridging molecules between PS on the apoptotic cell surface and PS recognition receptors on the phagocyte surface [104].

β2GPI, a well-known phospholipid-binding molecule [105, 106], is expressed by hepatocytes, endothelial cells and placental villous tissues [107]. It can bind to PS-exposing targets and help their interaction with macrophages through the generation of a specific bridging moiety [108].

C1q is the first component of the complement cascade pathway, which is part of the innate immune system. Unlike most complement proteins, which are produced by hepatocytes, C1q is mainly produced by macrophages [109]. C1q binding to PS mediates opsonization and phagocytosis of apoptotic cell debris and other PS-exposing targets, playing a crucial role in regulation of the immune response [110–114]. In addition, C1q has been shown to slow atherosclerosis progression by promoting macrophage survival and foam cell efferocytotic capacity in the early phases of atherosclerosis [115, 116].

#### Biological functions of PS recognition by receptors of CD300 family

Receptors of the CD300 family are type I transmembrane proteins that contain a single IgV-like extracellular domain with two disulfide bonds and intracellular immunoreceptor tyrosine-based inhibition motifs (ITIMs) [117]. Among the seven members of this family, only three CD300 molecules (i.e., CD300a, CD300b, and CD300f) have the ability to recognize PS exposed on the outer leaflet of activated cell membranes [118–120].

CD300a is expressed by myeloid cells [121], lymphoid cells, monocytes, macrophages, mast cells, granulocytes, DCs, NK cells and subsets of B and T cells [121]. Importantly, CD300a does not seem to be involved in efferocytosis. Its main function is the transduction of an inhibitory signal in mast cells leading to the reduced production of pro-inflammatory mediators [121].

CD300f is commonly expressed by myeloid cell lineages and increases myeloid cell efferocytotic ability [122]. In addition, it exerts an immunoregulatory function by inhibiting DC-mediated antigen-specific T-cell responses [123].

Both CD300a and CD300c may promote viral infections either by facilitating the binding between PS-containing viral particles and host cells or by easing viral escape mechanisms [124]. Noteworthy, these receptors have demonstrated great potential as therapeutic targets in the treatment of different diseases, including cancer, infectious diseases, allergies and other pathological conditions [118].

#### Biological functions of PS recognition by BAI1, LOX-1 and stabilin1/2

BAI1 is a transmembrane protein and a member of the adhesion-type G-protein-coupled receptor family with the ability of binding to PS via thrombospondin type 1 repeats. BAI1 is expressed in macrophages, myoblasts, glial and neuronal cells. It promotes the engulfment of apoptotic cells by forming a complex with engulfment and cell motility (ELMO)/dedicator of cytokinesis 1 (Dock180)/Rac and participating in the uptake process via actin cytoskeleton remodeling [125, 126]. In addition, under physiological conditions BAI1 promotes mammalian myogenesis by facilitating the myoblast fusion process [127].

LOX-1 is a type II membrane protein with a C-type lectin-like domain. It shows the ability to bind to various ligands, including modified lipoproteins [e.g., oxidized low-density lipoproteins (oxLDLs), acetylated low-density lipoproteins (acLDLs)], negatively charged phospholipids [e.g., PS and phosphatidylinositol (PI)] [128] and other ligands expressed by apoptotic cells, activated platelets and bacteria [129]. LOX-1 promotes efferocytosis by mediating the recognition of PS-containing apoptotic bodies [11, 130]. Importantly, LOX-1 also acts as a scavenger receptor mediating the uptake of oxLDLs by macrophages in atherosclerotic plaques [131, 132]. Accordingly, soluble LOX-1 (sLOX-1) has been suggested as a biomarker of cardiovascular risk and LOX-1 receptor blockade has been proposed as a potential therapeutic target for reduction of cardiovascular damage in systemic lupus erythematosus [132].

Stabilin-1 and stabilin-2 are multifunctional receptors, which share structural similarities but have significant functional differences. Structurally, stabilin-1 is a type-1 transmembrane receptor with a short cytoplasmic tail [133] and a scarce ligand repertoire. It is expressed in macrophages and in non-continuous sinusoidal endothelial cells of liver [134], spleen, lymph nodes and adrenal cortex [135–137]. The involvement of stabilin-1 in direct cell-cell communications appears to be crucial for cell migration [133], tissue homeostasis [138], and tumor development [139]. Stabilin-1-expressing macrophages have a pivotal role in maintaining tissue homeostasis and protecting against organ fibrosis in chronic liver injury [140]. In addition, stabilin-1 expression on macrophages contributes to the induction of an immunosuppressive profile in normal pregnancy of humans and to the maintenance of vascular integrity through the clearance of infected apoptotic endothelial cells in sepsis [141–143]. Finally, a stabilin-1-mediated pro-atherogenic effect has been suggested, as stabilin-1-expressing circulating monocytes of patients with familial hypercholesterolemia (FH) have shown increased CD36-mediated uptake of oxLDL [133]. Stabilin-2 is highly expressed in non-continuous sinusoidal endothelium of spleen, liver [134], lymph nodes and bone marrow [144] but shows restricted expression on a few macrophages including alveolar macrophages [138], and human monocyte-derived macrophages (HMDMs) [145]. Unlike stabilin-1, stabilin-2 seems to be a proper clearance receptor for hyaluronic acid (HA) on sinusoidal endothelial cells in the liver and a scavenger receptor for modified unwanted-self products [133, 135, 146]. Given the inhibitory action of HA in tumor cell metastasis, stabilin-2 inhibition, leading to elevated circulating HA levels, has been suggested as a potential antitumor strategy [147].

#### Biological functions of PS recognition by MFG-E8

MFG-E8 is a secreted glycoprotein which shows structural similarity to the coagulation factors V and VIII. Its second EGF-like domain consists of an RGD motif with the ability to bind to integrin αVβ3/5 in phagocytes [148]. MFG-E8 is broadly expressed in different organs and tissues (e.g., spleen, liver, lungs, kidneys, intestine, and mammary glands) by macrophages, DCs, fibroblasts, epithelial cells and osteoclasts [149, 150]. Integrin-binding activity is essential for a wide variety of MFG-E8-mediated efferocytosis-dependent/independent biological functions [151]. MFG-E8 inhibits neutrophil migration through αVβ3-integrin-mediated MAP kinase activation [152]. MFG-E8 also promotes macrophage M2 polarization in the tumor microenvironment, thereby promoting local immune suppression and facilitating tumor progression and metastasis [153, 154]. Consistent with MFG-E8-mediated anti-inflammatory activity, reduced MFG-E8 levels have been associated with an increased incidence of microvascular complications in patients with type 2 diabetes [155]. A variable association between MFG-E8 expression levels and autoimmune diseases has been described [156]. Accordingly, MFG-E8 is considered as a protective factor in the pathogenesis of rheumatoid arthritis [157], while high serum MFG-E8 levels or abnormally highly glycosylated serum MFG-E8 levels have been reported in some systemic lupus erythematosus patients [156, 158]. Septic shock is promoted by reduced serum levels of MFG-E8, resulting in defective efferocytosis [159]. Further**,** MFG-E8 deficiency in macrophages has been associated with reduced phagocytic clearance of apoptotic cells within atherosclerotic plaques, promoting atherosclerosis progression [160]. Accordingly, a genome-wide association meta-analysis showed that *MFGE8* as a contributory gene of coronary artery disease [161]. Finally, the ability of some enveloped viruses to infect integrin- and TAM receptor-presenting cells has been reported to be facilitated through the surface expression of MFG-E8 and Gas6 [162].

#### Biological functions of PS recognition by PSR

Using an established monoclonal antibody (i.e., mAb 217) binding both human and mouse macrophages and inhibiting the engulfment of apoptotic cells, the identification of a PS-binding membrane protein, that is, PSR, was prompted [163]. PSR, also named Jumonji domain-containing protein 6 (JMJD6), is a type II membrane protein expressed on macrophages, epithelial cells and fibroblasts [163]. Unlike other PS recognition receptors, PSR shows a low phospholipid-binding affinity and specificity for PS [164]. PSR-mediated phagocytosis has a crucial role in the maintenance of tissue homeostasis [165] and in regulation of the immune response [166]. PSR regulates the recognition and internalization of apoptotic photoreceptors and the conservation of retinal tissue architecture after retinal detachment [167]. Moreover, in central retinal vein occlusion (CRVO) red blood cell adhesion is facilitated by the interaction between PS RBC and endothelial PS receptor [168]. The clearance of PS-exposing particles present in the vascular wall, which is mediated by PSR, is important for the prevention of inflammation associated with necrosis, calcification and also elimination of thrombogenic factors. However, some studies revealed that PSR is also crucial for tissue remodeling and differentiation of various organs during embryogenesis through efferocytosis-independent molecular pathways [169–171]. In fact, homomultimers of PSR may function as scaffolding nuclear proteins with histone arginine demethylase activity regulating gene expression [172–178]. The upregulation of PSR has been described as an oncogenic driver in some tumor types [175, 176, 179, 180].

#### Biological functions of PS recognition by RAGE

RAGE is a transmembrane receptor of the immunoglobulin superfamily which binds to advanced glycation end products (AGEs) [181, 182]. RAGE activation has a crucial role in the pathogenesis of diabetic vascular complications [183–185], diabetic dyslipidemia [186] and diabetic nephropathy [187, 188]. In fact, AGE/RAGE signaling stimulates the production of reactive oxygen species (ROS) and inflammatory markers [189, 190]. In addition, the ligation of RAGE is one of the major means by which AGEs may impair cholesterol efflux and reverse cholesterol transport (RCT). Accordingly, RAGE binding to AGEs has been shown to suppress ATP-binding cassette sub-family G member 1 (ABCG1) and ATP-binding cassette transporter A1 (ABCA1) expression by macrophages. Also, RAGE activation has been associated with reduced circulating HDL levels in diabetic mice [186]. Accordingly, the regulation of AGE/RAGE signaling by miRNAs has been investigated as a therapeutic strategy against diabetes complications [191].

However, as a multiligand receptor, RAGE can also bind to PS and exert, like other PS recognition receptors, both efferocytosis-dependent and efferocytosis-independent biological functions. Accordingly, RAGE has been reported to modulate alveolar macrophage phagocytosis [192] and its dysfunction has been implicated in the abnormal remodeling of alveolar epithelium occurring in the pathogenesis of lung fibrosis [193]. In addition, RAGE has been shown to affect the expression of cell cycle genes modulating the G1/S phase transition [194, 195] and to stimulate phosphoinositide 3-kinase (PI3K)/protein kinase B (Akt) signaling pathway activation [196], thereby playing a crucial role in the development and progression of a number of tumor types [197].

### Phosphatidylethanolamine: as functional as PS or not?

Under certain conditions, including apoptosis, tumor-related angiogenesis, infections, and blood coagulation, loss of asymmetry of the plasma membrane of different cell types is observed, due to diminished activity of flippases and reduced transport of both PS and PE to the cytosolic face of the cell membrane [198].

Emoto and colleagues presented for the first time direct evidence that both PE and PS are externalized on the cell membrane surface during the early stages of apoptosis [199]. It is likely that PE exposure may promote apoptosis. Indeed, exogenous PE was reported to induce apoptosis in human hepatoma HepG2 cells through activation of the bcl-2/bax pathway [200]. In addition, Umeda and Emoto showed that the transbilayer PE redistribution in the plasma membrane was increased in apoptotic blebs, suggesting a role of PE in the reorganization of cytoskeletal structures during apoptosis [201]. However, the role of PE in efferocytosis is controversial and needs to be further explored. In this regard, a number of studies indicate that besides PS, PE can also act as a ligand for CD300a on the surface of phagocytes. However, the interaction between PE-exposing apoptotic cells and CD300a on phagocytes down-regulates the removal of apoptotic cells [120, 202]. In addition, another PS receptor involved in the regulation of phagocyte-mediated removal of dying cells, that is, Gas6, does not show any ability to bind to PE, suggesting the hypothesis that PE, unlike PS, does not have a crucial role in efferocytosis [54].

Several lines of evidence show that PE exposure on the cell surface is involved in a number of additional cell biological events apart from apoptosis and efferocytosis. Thus, for instance, PE expression on the outer face of the cell membrane is increased at the surface of the cleavage furrow which forms between two mitotic daughter cells and has a crucial role in the dynamics of contractile ring formation. PE redistribution from the inner to the outer leaflet of the membrane of endothelial cells is a feature of tumor vasculature in and around hypoxic areas, suggesting that PE could hold promise as a target for anti-tumor drugs and as a biomarker for tumor imaging [203]. There is evidence showing that PS exposure has a crucial role in certain infections. Indeed, recognition of PE-exposing viruses by two PS receptors (i.e., TIM-1 and TIM-4) has a pivotal role in the immune response against infections by numerous pathogenic viruses, including Ebola, West Nile and dengue viruses. Also, PE expression on the surface of intestinal epithelial cells may promote infection by enterohemorrhagic *Escherichia coli* (EHEC) [204]. Therefore, PE might be used as a broad-spectrum antimicrobial target [205, 206]. In addition, PE may enhance the cell membrane disruption by prefibrillar islet amyloid polypeptide protein (IAPP), an amyloidogenic protein. Indeed, although PE hampers the interaction of prefibrillar IAPP with cell membranes, it promotes IAPP-mediated cytotoxicity by favoring the growth of fibers on the membrane surface via a detergent-like mechanism [207]. Moreover, PE exposure by endothelial cells is involved in activation of the protein C anticoagulant pathway [208]. Finally, there are some studies reporting the ability of PE to interact with annexins within cell membranes, which may represent a unique model of regulation of different biological events [209].

### Concluding remarks

Apoptotic cell removal by phagocytes requires close collaboration between apoptotic cells and phagocytes. At the early stages of apoptosis, dying cells expose PS as an “eat me” signal. Subsequently, various receptors expressed by phagocytes, which can bind PS either directly or indirectly, promote apoptotic cell engulfment. Notably, accumulating evidence has elucidated the molecular mechanisms of PS externalization and the role of PS recognition receptors, their subunit structures, and their signaling pathways, including in efferocytosis-independent biological processes. Although extensive studies by several groups have greatly improved knowledge on multiple physiological functions of PS recognition receptors, some unanswered questions about the role of PS receptors in different pathological conditions need more investigations in order to fine-tune potential therapeutic strategies targeting these molecules.

Although PS has been widely studied, much less information is available about the function of PE exposure in apoptosis and efferocytosis, as well as other cellular processes. This might be partly due to the lack of particular detection systems with ability to discriminate between PE, PS or other phospholipids. However, the development of PE-specific probes allowing for the molecular imaging of cell death and other biological processes both in vitro and in vivo is expected to help unravel the specific role of PE exposure on the cell surface.

## Data Availability

Not applicable.

## Abbreviations

ABCA1: ATP-binding cassette transporter A1
ABCG1: ATP-binding cassette sub-family G member 1
acLDLs: acetylated low-density lipoprotein
AGEs: Advanced glycation end products
Akt: Protein kinase B
BAI1: Brain-specific angiogenesis inhibitor 1
C1q: Complement component 1q
CRVO: Central retinal vein occlusion
DCs: Dendritic cells
Dock180: Dedicator of cytokinesis 1
ELMO: Engulfment and cell motility
ERK: Extracellular signal-regulated kinase
FH: Familial hypercholesterolemia
Gas6: Growth arrest-specific gene 6
HA: Hyaluronic acid
HMDM: Human monocyte-derived macrophage
ICAM-3: Intercellular adhesion molecule-3
ITIMs: Immunoreceptor tyrosine-based inhibition motifs
JMJD6: Jumonji domain–containing protein 6
KIM-1: kidney injury molecule-1
LOX-1: Lectin-like oxidized low-density lipoprotein receptor-1
MAP: Mitogen-activated protein
MAPK: Mitogen-activated protein kinase
MFG-E8: Milk fat globule EGF factor 8
NK: Natural killer
oxLDL: oxidized low-density lipoprotein
PCR: Polymerase chain reaction
PE: Phosphatidylethanolamine
PI: Phosphatidylinositol
PI3K: Phosphoinositide 3-kinase
ProS: Protein S
PS: Phosphatidylserine
PSR: PS receptor
PTC: Proximal tubular cell
RAGE: Receptor for advanced glycosylation end products
RCT: Reverse cholesterol transport
ROS: Reactive oxygen species
RTKs: Receptor tyrosine kinases
sLOX-1: soluble LOX-1
TGF-β: Tumor growth factor-β
TIM: Transmembrane immunoglobulin and mucin domain
VSMC: Vascular smooth muscle cell
β2GPI: β2-glycoprotein I

## References

[1] Henson PM, Hume DA (2006). Apoptotic cell removal in development and tissue homeostasis. Trends Immunol.

[2] Nauta AJ, Daha MR, van Kooten C, Roos A (2003). Recognition and clearance of apoptotic cells: a role for complement and pentraxins. Trends Immunol.

[3] Gheibi Hayat SM, Bianconi V, Pirro M, Sahebkar A (2019). Efferocytosis: molecular mechanisms and pathophysiological perspectives. Immunol Cell Biol.

[4] Nagata S, Suzuki J, Segawa K, Fujii T (2016). Exposure of phosphatidylserine on the cell surface. Cell Death Differ.

[5] Ravichandran KS (2011). Beginnings of a good apoptotic meal: the find-me and eat-me signaling pathways. Immunity.

[6] Segawa K, Nagata S (2015). An apoptotic ‘eat me’signal: phosphatidylserine exposure. Trends Cell Biol.

[7] Medina C, Ravichandran K (2016). Do not let death dous part:‘find-me’signals in communication between dying cells and the phagocytes. Cell Death Differ.

[8] Birge R, Boeltz S, Kumar S, Carlson J, Wanderley J, Calianese D (2016). Phosphatidylserine is a global immunosuppressive signal in efferocytosis, infectious disease, and cancer. Cell Death Differ.

[9] Penberthy KK, Ravichandran KS (2016). Apoptotic cell recognition receptors and scavenger receptors. Immunol Rev.

[10] Martin S, Reutelingsperger C, McGahon AJ, Rader JA, Van Schie R, LaFace DM (1995). Early redistribution of plasma membrane phosphatidylserine is a general feature of apoptosis regardless of the initiating stimulus: inhibition by overexpression of Bcl-2 and Abl. J Exp Med.

[11] Murphy JE, Tacon D, Tedbury PR, Hadden JM, Knowling S, Sawamura T (2006). LOX-1 scavenger receptor mediates calcium-dependent recognition of phosphatidylserine and apoptotic cells. Biochem J.

[12] Schoenwaelder SM, Yuan Y, Josefsson EC, White MJ, Yao Y, Mason KD (2009). Two distinct pathways regulate platelet phosphatidylserine exposure and procoagulant function. Blood.

[13] Nagata S (2018). Apoptosis and clearance of apoptotic cells. Annu Rev Immunol.

[14] Krahling S, Callahan MK, Williamson P, Schlegel RA (1999). Exposure of phosphatidylserine is a general feature in the phagocytosis of apoptotic lymphocytes by macrophages. Cell Death Differ.

[15] Asano K, Miwa M, Miwa K, Hanayama R, Nagase H, Nagata S (2004). Masking of phosphatidylserine inhibits apoptotic cell engulfment and induces autoantibody production in mice. J Exp Med.

[16] Arandjelovic S, Ravichandran KS (2015). Phagocytosis of apoptotic cells in homeostasis. Nat Immunol.

[17] Arur S, Uche UE, Rezaul K, Fong M, Scranton V, Cowan AE (2003). Annexin I is an endogenous ligand that mediates apoptotic cell engulfment. Dev Cell.

[18] Gardai SJ, McPhillips KA, Frasch SC, Janssen WJ, Starefeldt A, Murphy-Ullrich JE (2005). Cell-surface calreticulin initiates clearance of viable or apoptotic cells through trans-activation of LRP on the phagocyte. Cell.

[19] Oldenborg P-A, Zheleznyak A, Fang Y-F, Lagenaur CF, Gresham HD, Lindberg FP (2000). Role of CD47 as a marker of self on red blood cells. Science.

[20] Brown S, Heinisch I, Ross E, Shaw K, Buckley CD, Savill J (2002). Apoptosis disables CD31-mediated cell detachment from phagocytes promoting binding and engulfment. Nature.

[21] Gardai SJ, Bratton DL, Ogden CA, Henson PM (2006). Recognition ligands on apoptotic cells: a perspective. J Leukoc Biol.

[22] Riedl S, Rinner B, Asslaber M, Schaider H, Walzer S, Novak A (2011). In search of a novel target—phosphatidylserine exposed by non-apoptotic tumor cells and metastases of malignancies with poor treatment efficacy. Biochim Biophys Acta.

[23] Sharma B, Kanwar SS. Phosphatidylserine: A cancer cell targeting biomarker. Semin Cancer Biol. 2018;52(Pt 1):17–25.10.1016/j.semcancer.2017.08.01228870843

[24] Nagata S, Hanayama R, Kawane K (2010). Autoimmunity and the clearance of dead cells. Cell.

[25] Abdolmaleki F, Farahani N, Gheibi Hayat SM, Pirro M, Bianconi V, Barreto GE (2018). The role of Efferocytosis in autoimmune diseases. Front Immunol.

[26] Tajbakhsh A, Bianconi V, Pirro M, Gheibi Hayat SM, Johnston TP, Sahebkar A (2019). Efferocytosis and atherosclerosis: regulation of phagocyte function by MicroRNAs. Trends Endocrinol Metab.

[27] Tajbakhsh A, Gheibi Hayat SM, Butler AE, Sahebkar A (2019). Effect of soluble cleavage products of important receptors/ligands on efferocytosis: their role in inflammatory, autoimmune and cardiovascular disease. Ageing Res Rev.

[28] Tajbakhsh A, Rezaee M, Kovanen PT, Sahebkar A (2018). Efferocytosis in atherosclerotic lesions: malfunctioning regulatory pathways and control mechanisms. Pharmacol Ther.

[29] Abu-Baker S, Chu Z, Stevens AM, Li J, Qi X (2012). Cytotoxicity and selectivity in skin cancer by SapC-DOPS nanovesicles. J Cancer Ther.

[30] Davis HW, Hussain N, Qi X (2016). Detection of cancer cells using SapC-DOPS nanovesicles. Mol Cancer.

[31] Chu Z, Abu-Baker S, Palascak MB, Ahmad SA, Franco RS, Qi X (2013). Targeting and cytotoxicity of SapC-DOPS nanovesicles in pancreatic cancer. PLoS One.

[32] Heemskerk JW, Bevers EM, Lindhout T (2002). Platelet activation and blood coagulation. Thromb Haemost.

[33] Ehlen HW, Chinenkova M, Moser M, Munter HM, Krause Y, Gross S (2013). Inactivation of anoctamin-6/Tmem16f, a regulator of phosphatidylserine scrambling in osteoblasts, leads to decreased mineral deposition in skeletal tissues. J Bone Miner Res.

[34] van den Eijnde SM, van den Hoff MJ, Reutelingsperger CP, van Heerde WL, Henfling ME, Vermeij-Keers C (2001). Transient expression of phosphatidylserine at cell-cell contact areas is required for myotube formation. J Cell Sci.

[35] Nanbo A, Kawaoka Y (2019). Molecular mechanism of externalization of phosphatidylserine on the surface of Ebola virus particles. DNA Cell Biol.

[36] Abay ZC, Wong MY-Y, Teoh J-S, Vijayaraghavan T, Hilliard MA, Neumann B (2017). Phosphatidylserine save-me signals drive functional recovery of severed axons in Caenorhabditis elegans. Proc Natl Acad Sci.

[37] Adler RR, Ng A-K, Rote NS (1995). Monoclonal antiphosphatidylserine antibody inhibits intercellular fusion of the choriocarcinoma line, JAR. Biol Reprod.

[38] Callahan M, Williamson P, Schlegel R (2000). Surface expression of phosphatidylserine on macrophages is required for phagocytosis of apoptotic thymocytes. Cell Death Differ.

[39] Helming L, Winter J, Gordon S (2009). The scavenger receptor CD36 plays a role in cytokine-induced macrophage fusion. J Cell Sci.

[40] Dowall S, Graham V, Corbin-Lickfett K, Empig C, Schlunegger K, Bruce C, et al. Effective binding of a phosphatidylserine-targeting antibody to Ebola virus infected cells and purified virions. J Immunol Res. 2015;2015:347903. 10.1155/2015/347903.10.1155/2015/347903PMC435980625815346

[41] Meertens L, Carnec X, Lecoin MP, Ramdasi R, Guivel-Benhassine F, Lew E (2012). The TIM and TAM families of phosphatidylserine receptors mediate dengue virus entry. Cell Host Microbe.

[42] Moller-Tank S, Kondratowicz AS, Davey RA, Rennert PD, Maury W (2013). Role of the phosphatidylserine receptor TIM-1 in enveloped-virus entry. J Virol.

[43] Elkon KB, Silverman GJ. Naturally occurring autoantibodies to apoptotic cells. Naturally Occurring Antibodies (NAbs). Adv Exp Med Biol. 2012;750:14–26.10.1007/978-1-4614-3461-0_222903663

[44] Fernandez-Arias C, Rivera-Correa J, Gallego-Delgado J, Rudlaff R, Fernandez C, Roussel C (2016). Anti-self phosphatidylserine antibodies recognize uninfected erythrocytes promoting malarial anemia. Cell Host Microbe.

[45] Hayat SMG, Bianconi V, Pirro M, Jaafari MR, Hatamipour M, Sahebkar A (2020). CD47: role in the immune system and application to cancer therapy. Cell Oncol.

[46] Kim R, Emi M, Tanabe K, Arihiro K (2006). Tumor-driven evolution of immunosuppressive networks during malignant progression. Cancer Res.

[47] Arthur CM, Rodrigues LC, Baruffi MD, Sullivan HC, Cummings RD, Stowell SR (2015). Detection of phosphatidylserine exposure on leukocytes following treatment with human galectins.

[48] Fischer K, Voelkl S, Berger J, Andreesen R, Pomorski T, Mackensen A (2006). Antigen recognition induces phosphatidylserine exposure on the cell surface of human CD8+ T cells. Blood.

[49] Stowell SR, Karmakar S, Arthur CM, Ju T, Rodrigues LC, Riul TB (2009). Galectin-1 induces reversible phosphatidylserine exposure at the plasma membrane. Mol Biol Cell.

[50] Rothlin CV, Carrera-Silva EA, Bosurgi L, Ghosh S (2015). TAM receptor signaling in immune homeostasis. Annu Rev Immunol.

[51] Graham DK, Dawson TL, Mullaney DL, Snodgrass HR, Earp HS (1994). Cloning and mRNA expression analysis of a novel human protooncogene, c-mer. Cell Growth Differ.

[52] Polvi A, Armstrong E, Lai G, Lemke G, Huebner K, Spritz RA (1993). The human TYROS gene and pseudogene are located in chromosome 15q14-q25. Gene.

[53] Benzakour O, Gely A, Lara R, Coronas V (2007). Gas-6 and protein S: vitamin K-dependent factors and ligands for the TAM tyrosine kinase receptors family. Med Sci.

[54] Nakano T, Ishimoto Y, Kishino J, Umeda M, Inoue K, Nagata K (1997). Cell adhesion to phosphatidylserine mediated by a product of growth arrest-specific gene 6. J Biol Chem.

[55] Anderson HA, Maylock CA, Williams JA, Paweletz CP, Shu H, Shacter E (2003). Serum-derived protein S binds to phosphatidylserine and stimulates the phagocytosis of apoptotic cells. Nat Immunol.

[56] Ravichandran KS (2010). Find-me and eat-me signals in apoptotic cell clearance: progress and conundrums. J Exp Med.

[57] Zagórska A, Través PG, Lew ED, Dransfield I, Lemke G (2014). Diversification of TAM receptor tyrosine kinase function. Nat Immunol.

[58] Hafizi S, Dahlbäck B (2006). Signalling and functional diversity within the Axl subfamily of receptor tyrosine kinases. Cytokine Growth Factor Rev.

[59] Yanagihashi Y, Segawa K, Maeda R (2017). Nabeshima Y-i, Nagata S. mouse macrophages show different requirements for phosphatidylserine receptor Tim4 in efferocytosis. Proc Natl Acad Sci.

[60] Lemke G (2013). Biology of the TAM receptors. Cold Spring Harb Perspect Biol.

[61] Lemke G (2017). Phosphatidylserine is the signal for TAM receptors and their ligands. Trends Biochem Sci.

[62] Cosemans J, Van Kruchten R, Olieslagers S, Schurgers L, Verheyen F, Munnix I (2010). Potentiating role of Gas6 and Tyro3, Axl and Mer (TAM) receptors in human and murine platelet activation and thrombus stabilization. J Thromb Haemost.

[63] Gjerdrum C, Tiron C, Høiby T, Stefansson I, Haugen H, Sandal T (2010). Axl is an essential epithelial-to-mesenchymal transition-induced regulator of breast cancer metastasis and patient survival. Proc Natl Acad Sci.

[64] Dunne PD, McArt DG, Blayney JK, Kalimutho M, Greer S, Wang T (2014). AXL is a key regulator of inherent and chemotherapy-induced invasion and predicts a poor clinical outcome in early-stage colon cancer. Clin Cancer Res.

[65] Rothlin CV, Ghosh S, Zuniga EI, Oldstone MB, Lemke G (2007). TAM receptors are pleiotropic inhibitors of the innate immune response. Cell.

[66] Graham DK, DeRyckere D, Davies KD, Earp HS (2014). The TAM family: phosphatidylserine-sensing receptor tyrosine kinases gone awry in cancer. Nat Rev Cancer.

[67] Lew ED, Oh J, Burrola PG, Lax I, Zagórska A, Través PG (2014). Differential TAM receptor–ligand–phospholipid interactions delimit differential TAM bioactivities. Elife.

[68] Stanford JC, Young C, Hicks D, Owens P, Williams A, Vaught DB (2014). Efferocytosis produces a prometastatic landscape during postpartum mammary gland involution. J Clin Invest.

[69] Bozic I, Reiter JG, Allen B, Antal T, Chatterjee K, Shah P (2013). Evolutionary dynamics of cancer in response to targeted combination therapy. elife.

[70] Bosurgi L, Bernink JH, Cuevas VD, Gagliani N, Joannas L, Schmid ET (2013). Paradoxical role of the proto-oncogene Axl and Mer receptor tyrosine kinases in colon cancer. Proc Natl Acad Sci.

[71] Dransfield I, Zagórska A, Lew E, Michail K, Lemke G (2016). Mer receptor tyrosine kinase mediates both tethering and phagocytosis of apoptotic cells. Cell Death Dis.

[72] Lu Q, Lemke G (2001). Homeostatic regulation of the immune system by receptor tyrosine kinases of the tyro 3 family. Science.

[73] Scott RS, McMahon EJ, Pop SM, Reap EA, Caricchio R, Cohen PL (2001). Phagocytosis and clearance of apoptotic cells is mediated by MER. Nature.

[74] Cohen PL, Caricchio R, Abraham V, Camenisch TD, Jennette JC, Roubey RA (2002). Delayed apoptotic cell clearance and lupus-like autoimmunity in mice lacking the c-mer membrane tyrosine kinase. J Exp Med.

[75] Thorp E, Vaisar T, Subramanian M, Mautner L, Blobel C, Tabas I (2011). Shedding of the Mer tyrosine kinase receptor is mediated by ADAM17 protein through a pathway involving reactive oxygen species, protein kinase Cδ, and p38 mitogen-activated protein kinase (MAPK). J Biol Chem.

[76] Cai B, Thorp EB, Doran AC, Sansbury BE, Daemen MJ, Dorweiler B (2017). MerTK receptor cleavage promotes plaque necrosis and defective resolution in atherosclerosis. J Clin Invest.

[77] Thorp E, Cui D, Schrijvers DM, Kuriakose G, Tabas I (2008). Mertk receptor mutation reduces efferocytosis efficiency and promotes apoptotic cell accumulation and plaque necrosis in atherosclerotic lesions of apoe−/− mice. Arterioscler Thromb Vasc Biol.

[78] Ming Cao W, Murao K, Imachi H, Sato M, Nakano T, Kodama T (2001). Phosphatidylinositol 3-OH kinase–Akt/protein kinase B pathway mediates Gas6 induction of scavenger receptor a in immortalized human vascular smooth muscle cell line. Arterioscler Thromb Vasc Biol.

[79] Tjwa M, Bellido-Martin L, Lin Y, Lutgens E, Plaisance S, Bono F (2008). Gas6 promotes inflammation by enhancing interactions between endothelial cells, platelets, and leukocytes. Blood.

[80] Freeman GJ, Casasnovas JM, Umetsu DT, DeKruyff RH (2010). TIM genes: a family of cell surface phosphatidylserine receptors that regulate innate and adaptive immunity. Immunol Rev.

[81] Miyanishi M, Tada K, Koike M, Uchiyama Y, Kitamura T, Nagata S (2007). Identification of Tim4 as a phosphatidylserine receptor. Nature.

[82] Brooks CR, Bonventre JV (2015). KIM-1/TIM-1 in proximal tubular cell immune response. Oncotarget.

[83] Yin W, Naini SM, Chen G, Hentschel DM, Humphreys BD, Bonventre JV (2016). Mammalian target of rapamycin mediates kidney injury molecule 1-dependent tubule injury in a surrogate model. J Am Soc Nephrol.

[84] Ichimura T, Asseldonk EJ, Humphreys BD, Gunaratnam L, Duffield JS, Bonventre JV (2008). Kidney injury molecule–1 is a phosphatidylserine receptor that confers a phagocytic phenotype on epithelial cells. J Clin Invest.

[85] Yang L, Brooks CR, Xiao S, Sabbisetti V, Yeung MY, Hsiao L-L (2015). KIM-1–mediated phagocytosis reduces acute injury to the kidney. J Clin Invest.

[86] Bonventre JV (2014). Kidney injury molecule-1: a translational journey. Trans Am Clin Climatol Assoc.

[87] Ajay AK, Kim T-M, Ramirez-Gonzalez V, Park PJ, Frank DA, Vaidya VS (2014). A bioinformatics approach identifies signal transducer and activator of transcription-3 and checkpoint kinase 1 as upstream regulators of kidney injury molecule-1 after kidney injury. J Am Soc Nephrol.

[88] Askenazi DJ, Koralkar R, Levitan EB, Goldstein SL, Devarajan P, Khandrika S (2011). Baseline values of candidate urine acute kidney injury biomarkers vary by gestational age in premature infants. Pediatr Res.

[89] Han WK, Bailly V, Abichandani R, Thadhani R, Bonventre JV (2002). Kidney injury Molecule-1 (KIM-1): a novel biomarker for human renal proximal tubule injury. Kidney Int.

[90] van Timmeren MM, van den Heuvel MC, Bailly V, Bakker SJ, van Goor H, Stegeman CA (2007). Tubular kidney injury molecule-1 (KIM-1) in human renal disease. J Pathol.

[91] Ismail OZ, Zhang X, Wei J, Haig A, Denker BM, Suri RS (2015). Kidney injury molecule-1 protects against Gα12 activation and tissue damage in renal ischemia-reperfusion injury. Am J Pathol.

[92] Zhang Z, Cai CX (2016). Kidney injury molecule-1 (KIM-1) mediates renal epithelial cell repair via ERK MAPK signaling pathway. Mol Cell Biochem.

[93] Wong SH, Barlow JL, Nabarro S, Fallon PG, McKenzie AN (2010). Tim-1 is induced on germinal Centre B cells through B-cell receptor signalling but is not essential for the germinal Centre response. Immunology.

[94] Rennert PD (2011). Novel roles for TIM-1 in immunity and infection. Immunol Lett.

[95] Brooks CR, Yeung MY, Brooks YS, Chen H, Ichimura T, Henderson JM (2015). KIM-1−/TIM-1-mediated phagocytosis links ATG5−/ULK1-dependent clearance of apoptotic cells to antigen presentation. EMBO J.

[96] Thornley TB, Fang Z, Balasubramanian S, Larocca RA, Gong W, Gupta S (2014). Fragile TIM-4–expressing tissue resident macrophages are migratory and immunoregulatory. J Clin Invest.

[97] Bonnardel J, Da Silva C, Henri S, Tamoutounour S, Chasson L, Montañana-Sanchis F (2015). Innate and adaptive immune functions of peyer’s patch monocyte-derived cells. Cell Rep.

[98] Park D, Hochreiter-Hufford A, Ravichandran KS (2009). The phosphatidylserine receptor TIM-4 does not mediate direct signaling. Curr Biol.

[99] Somersan S, Bhardwaj N (2001). Tethering and tickling: a new role for the phosphatidylserine receptor. J Cell Biol.

[100] Dorfman DM, Hornick JL, Shahsafaei A, Freeman GJ (2010). The phosphatidylserine receptors, T cell immunoglobulin mucin proteins 3 and 4, are markers of histiocytic sarcoma and other histiocytic and dendritic cell neoplasms. Hum Pathol.

[101] Zhang Q, Wang H, Wu X, Liu B, Liu W, Wang R (2015). TIM-4 promotes the growth of non-small-cell lung cancer in a RGD motif-dependent manner. Br J Cancer.

[102] Xu L, Xiao H, Xu M, Zhou C, Yi L, Liang H (2011). Glioma-derived T cell immunoglobulin-and mucin domain-containing molecule-4 (TIM4) contributes to tumor tolerance. J Biol Chem.

[103] Levine JS, Ucker DS (2019). Voices from the dead: the complex vocabulary and intricate grammar of dead cells. Adv Protein Chem Struct Biol.

[104] Rosenbaum S, Kreft S, Etich J, Frie C, Stermann J, Grskovic I (2011). Identification of novel binding partners (annexins) for the cell death signal phosphatidylserine and definition of their recognition motif. J Biol Chem.

[105] De Laat HB, Derksen RH, de Groot PG (2004). β2-glycoprotein I, the playmaker of the antiphospholipid syndrome. Clin Immunol.

[106] de Groot PG, Urbanus RT (2012). The significance of autoantibodies against β2-glycoprotein I. Blood.

[107] Caronti B, Calderaro C, Alessandri C, Conti F, Tinghino R, Palladini G (1999). β2-glycoprotein I (β2-GPI) mRNA is expressed by several cell types involved in anti-phospholipid syndrome-related tissue damage. Clin Exp Immunol.

[108] Balasubramanian K, Schroit AJ (1998). Characterization of phosphatidylserine-dependent β2-glycoprotein I macrophage interactions IMPLICATIONS FOR APOPTOTIC CELL CLEARANCE BY PHAGOCYTES. J Biol Chem.

[109] Petry F, Botto M, Holtappels R, Walport MJ, Loos M (2001). Reconstitution of the complement function in C1q-deficient (C1qa−/−) mice with wild-type bone marrow cells. J Immunol.

[110] Manderson AP, Botto M, Walport MJ (2004). The role of complement in the development of systemic lupus erythematosus. Annu Rev Immunol.

[111] Korb LC, Ahearn JM (1997). C1q binds directly and specifically to surface blebs of apoptotic human keratinocytes: complement deficiency and systemic lupus erythematosus revisited. J Immunol.

[112] Navratil JS, Watkins SC, Wisnieski JJ, Ahearn JM (2001). The globular heads of C1q specifically recognize surface blebs of apoptotic vascular endothelial cells. J Immunol.

[113] Gaboriaud C, Frachet P, Thielens N, Arlaud G (2012). The human c1q globular domain: structure and recognition of non-immune self ligands. Front Immunol.

[114] Nauta AJ, Trouw LA, Daha MR, Tijsma O, Nieuwland R, Schwaeble WJ (2002). Direct binding of C1q to apoptotic cells and cell blebs induces complement activation. Eur J Immunol.

[115] Pulanco MC, Cosman J, Ho M-M, Huynh J, Fing K, Turcu J (2017). Complement protein C1q enhances macrophage foam cell survival and efferocytosis. J Immunol.

[116] Bhatia VK, Yun S, Leung V, Grimsditch DC, Benson GM, Botto MB (2007). Complement C1q reduces early atherosclerosis in low-density lipoprotein receptor-deficient mice. Am J Pathol.

[117] Clark GJ, Ju X, Tate C, Hart DN (2009). The CD300 family of molecules are evolutionarily significant regulators of leukocyte functions. Trends Immunol.

[118] Borrego F (2013). The CD300 molecules: an emerging family of regulators of the immune system. Blood.

[119] Murakami Y, Tian L, Voss O, Margulies D, Krzewski K, Coligan J (2014). CD300b regulates the phagocytosis of apoptotic cells via phosphatidylserine recognition. Cell Death Differ.

[120] Simhadri VR, Andersen JF, Calvo E, Choi S-C, Coligan JE, Borrego F (2012). Human CD300a binds to phosphatidylethanolamine and phosphatidylserine, and modulates the phagocytosis of dead cells. Blood.

[121] Nakahashi-Oda C, Tahara-Hanaoka S, Honda S-I, Shibuya K, Shibuya A (2012). Identification of phosphatidylserine as a ligand for the CD300a immunoreceptor. Biochem Biophys Res Commun.

[122] Korver W, Zhao X, Singh S, Pardoux C, Zhao J, Guzman M (2009). Monoclonal antibodies against IREM-1: potential for targeted therapy of AML. Leukemia.

[123] Shi L, Luo K, Xia D, Chen T, Chen G, Jiang Y (2006). DIgR2, dendritic cell-derived immunoglobulin receptor 2, is one representative of a family of IgSF inhibitory receptors and mediates negative regulation of dendritic cell-initiated antigen-specific T-cell responses. Blood.

[124] Vitallé J, Terrén I, Orrantia A, Zenarruzabeitia O, Borrego F (2019). CD300 receptor family in viral infections. Eur J Immunol.

[125] Park D, Tosello-Trampont A-C, Elliott MR, Lu M, Haney LB, Ma Z (2007). BAI1 is an engulfment receptor for apoptotic cells upstream of the ELMO/Dock180/Rac module. Nature.

[126] Hermetet F, Jacquin E, Launay S, Gaiffe E, Couturier M, Hirchaud F (2016). Efferocytosis of apoptotic human papillomavirus-positive cervical cancer cells by human primary fibroblasts. Biol Cell.

[127] Hochreiter-Hufford AE, Lee CS, Kinchen JM, Sokolowski JD, Arandjelovic S, Call JA (2013). Phosphatidylserine receptor BAI1 and apoptotic cells as new promoters of myoblast fusion. Nature.

[128] Moriwaki H, Kume N, Sawamura T, Aoyama T, Hoshikawa H, Ochi H (1998). Ligand specificity of LOX-1, a novel endothelial receptor for oxidized low density lipoprotein. Arterioscler Thromb Vasc Biol.

[129] Mehta JL, Chen J, Hermonat PL, Romeo F, Novelli G (2006). Lectin-like, oxidized low-density lipoprotein receptor-1 (LOX-1): a critical player in the development of atherosclerosis and related disorders. Cardiovasc Res.

[130] Chen M, Masaki T, Sawamura T (2002). LOX-1, the receptor for oxidized low-density lipoprotein identified from endothelial cells: implications in endothelial dysfunction and atherosclerosis. Pharmacol Ther.

[131] Kakutani M, Masaki T, Sawamura T (2000). A platelet–endothelium interaction mediated by lectin-like oxidized low-density lipoprotein receptor-1. Proc Natl Acad Sci.

[132] Sagar D, Gaddipati R, Ongstad E, Rahman S, Belkhodja M, Bhagroo N, et al. Soluble LOX-1: a potential biomarker for SLE and cardiovascular comorbidity. J Immunol. 2018;200:S45.1.

[133] Kzhyshkowska J (2010). Multifunctional receptor stabilin-1 in homeostasis and disease. Sci World J.

[134] Schledzewski K, Géraud C, Arnold B, Wang S, Gröne H-J, Kempf T (2011). Deficiency of liver sinusoidal scavenger receptors stabilin-1 and-2 in mice causes glomerulofibrotic nephropathy via impaired hepatic clearance of noxious blood factors. J Clin Invest.

[135] Goerdt S, Walsh LJ, Murphy GF, Pober JS (1991). Identification of a novel high molecular weight protein preferentially expressed by sinusoidal endothelial cells in normal human tissues. J Cell Biol.

[136] Kzhyshkowska J, Gratchev A, Goerdt S (2006). Stabilin-1, a homeostatic scavenger receptor with multiple functions. J Cell Mol Med.

[137] Schönhaar K, Schledzewski K, Michel J, Dollt C, Gkaniatsou C, Géraud C (2014). Expression of stabilin-1 in M2 macrophages in human granulomatous disease and melanocytic lesions. Int J Clin Exp Pathol.

[138] Park S-Y, Jung M-Y, Lee S-J, Kang K-B, Gratchev A, Riabov V (2009). Stabilin-1 mediates phosphatidylserine-dependent clearance of cell corpses in alternatively activated macrophages. J Cell Sci.

[139] Riabov V, Yin S, Song B, Avdic A, Schledzewski K, Ovsiy I (2016). Stabilin-1 is expressed in human breast cancer and supports tumor growth in mammary adenocarcinoma mouse model. Oncotarget.

[140] Rantakari P, Patten DA, Valtonen J, Karikoski M, Gerke H, Dawes H (2016). Stabilin-1 expression defines a subset of macrophages that mediate tissue homeostasis and prevent fibrosis in chronic liver injury. Proc Natl Acad Sci.

[141] Palani S, Elima K, Ekholm E, Jalkanen S, Salmi M (2016). Monocyte stabilin-1 suppresses the activation of Th1 lymphocytes. J Immunol.

[142] Mosig S, Rennert K, Krause S, Kzhyshkowska J, Neunübel K, Heller R (2009). Different functions of monocyte subsets in familial hypercholesterolemia: potential function of CD14+ CD16+ monocytes in detoxification of oxidized LDL. FASEB J.

[143] Lee W, Park S-Y, Yoo Y, Kim S-Y, Kim J-E, Kim S-W (2018). Macrophagic Stabilin-1 restored disruption of vascular integrity caused by sepsis. Thromb Haemost.

[144] Rosie ZY, Kim T-W, Hong A, Watanabe TA, Gaus HJ, Geary RS (2007). Cross-species pharmacokinetic comparison from mouse to man of a second-generation antisense oligonucleotide, ISIS 301012, targeting human apolipoprotein B-100. Drug Metab Dispos.

[145] Park S, Jung M, Kim H, Lee S, Kim S, Lee B (2008). Rapid cell corpse clearance by stabilin-2, a membrane phosphatidylserine receptor. Cell Death Differ.

[146] Hansen B, Longati P, Elvevold K, Nedredal G-I, Schledzewski K, Olsen R (2005). Stabilin-1 and stabilin-2 are both directed into the early endocytic pathway in hepatic sinusoidal endothelium via interactions with clathrin/AP-2, independent of ligand binding. Exp Cell Res.

[147] Hirose Y, Saijou E, Sugano Y, Takeshita F, Nishimura S, Nonaka H (2012). Inhibition of Stabilin-2 elevates circulating hyaluronic acid levels and prevents tumor metastasis. Proc Natl Acad Sci.

[148] Hanayama R, Tanaka M, Miwa K, Shinohara A, Iwamatsu A, Nagata S (2002). Identification of a factor that links apoptotic cells to phagocytes. Nature.

[149] Aziz M, Jacob A, Matsuda A, Wang P (2011). milk fat globule-EGF factor 8 expression, function and plausible signal transduction in resolving inflammation. Apoptosis.

[150] Abe T, Shin J, Hosur K, Udey MC, Chavakis T, Hajishengallis G (2014). Regulation of osteoclast homeostasis and inflammatory bone loss by MFG-E8. J Immunol.

[151] Ooishi T, Nadano D, Matsuda T, Oshima K (2017). Extracellular vesicle-mediated MFG-E8 localization in the extracellular matrix is required for its integrin-dependent function in mouse mammary epithelial cells. Genes Cells.

[152] Aziz M, Yang WL, Corbo LM, Chaung WW, Matsuo S, Wang P (2015). MFG-E8 inhibits neutrophil migration through αvβ3-integrin-dependent MAP kinase activation. Int J Mol Med.

[153] Yamada K, Uchiyama A, Uehara A, Perera B, Ogino S, Yokoyama Y (2016). MFG-E8 drives melanoma growth by stimulating mesenchymal stromal cell-induced angiogenesis and M2 polarization of tumor-associated macrophages. Cancer Res.

[154] Jinushi M, Sato M, Kanamoto A, Itoh A, Nagai S, Koyasu S (2009). Milk fat globule epidermal growth factor–8 blockade triggers tumor destruction through coordinated cell-autonomous and immune-mediated mechanisms. J Exp Med.

[155] Sun G, Liu J, Xia G, Zhang L, Li Y, Zhou Z (2017). Reduced serum milk fat globule-epidermal growth factor 8 (MFG-E8) concentrations are associated with an increased risk of microvascular complications in patients with type 2 diabetes. Clin Chim Acta.

[156] Yamaguchi H, Takagi J, Miyamae T, Yokota S, Fujimoto T, Nakamura S (2008). Milk fat globule EGF factor 8 in the serum of human patients of systemic lupus erythematosus. J Leukoc Biol.

[157] Albus E, Sinningen K, Winzer M, Thiele S, Baschant U, Hannemann A (2016). Milk fat globule-epidermal growth factor 8 (MFG-E8) is a novel anti-inflammatory factor in rheumatoid arthritis in mice and humans. J Bone Miner Res.

[158] Yamaguchi H, Fujimoto T, Nakamura S, Ohmura K, Mimori T, Matsuda F (2010). Aberrant splicing of the milk fat globule-EGF factor 8 (MFG-E8) gene in human systemic lupus erythematosus. Eur J Immunol.

[159] Miksa M, Wu R, Dong W, Komura H, Amin D, Ji Y (2009). Immature dendritic cell-derived exosomes rescue septic animals via milk fat globule epidermal growth factor VIII. J Immunol.

[160] Ait-Oufella H, Kinugawa K, Zoll J, Simon T, Boddaert J, Heeneman S (2007). CLINICAL PERSPECTIVE. Circulation.

[161] Nikpay M, Goel A, Won H-H, Hall LM, Willenborg C, Kanoni S (2015). A comprehensive 1000 genomes–based genome-wide association meta-analysis of coronary artery disease. Nat Genet.

[162] Morizono K, Chen IS (2014). Role of phosphatidylserine receptors in enveloped virus infection. J Virol.

[163] Fadok VA, Bratton DL, Rose DM, Pearson A, Ezekewitz RAB, Henson PM (2000). A receptor for phosphatidylserine-specific clearance of apoptotic cells. Nature.

[164] Yang H, Chen Y-Z, Zhang Y, Wang X, Zhao X, Godfroy JI (2015). A lysine-rich motif in the phosphatidylserine receptorPSR-1 mediates recognition and removal of apoptotic cells. Nat Commun.

[165] Mitchell JE, Cvetanovic M, Tibrewal N, Patel V, Colamonici OR, Li MO (2006). The presumptive phosphatidylserine receptor is dispensable for innate anti-inflammatory recognition and clearance of apoptotic cells. J Biol Chem.

[166] Hoffmann PR, Kench JA, Vondracek A, Kruk E, Daleke DL, Jordan M (2005). Interaction between phosphatidylserine and the phosphatidylserine receptor inhibits immune responses in vivo. J Immunol.

[167] Hisatomi T, Sakamoto T, Sonoda K-H, Tsutsumi C, Qiao H, Enaida H (2003). Clearance of apoptotic photoreceptors: elimination of apoptotic debris into the subretinal space and macrophage-mediated phagocytosis via phosphatidylserine receptor and integrin αvβ3. Am J Pathol.

[168] Wautier J-L, Wautier M-P (2013). Molecular basis of erythrocyte adhesion to endothelial cells in diseases. Clin Hemorheol Microcirc.

[169] Böse J, Gruber AD, Helming L, Schiebe S, Wegener I, Hafner M (2004). The phosphatidylserine receptor has essential functions during embryogenesis but not in apoptotic cell removal. J Biol.

[170] Taung W-L, Wu J-L, Hong J-R (2018). The role of PSR in zebrafish (Danio rerio) at early embryonic development. Recent Advances in Zebrafish Researches: IntechOpen.

[171] Atkin-Smith GK, Poon IK (2017). Disassembly of the dying: mechanisms and functions. Trends Cell Biol.

[172] Klose RJ, Kallin EM, Zhang Y (2006). JmjC-domain-containing proteins and histone demethylation. Nat Rev Genet.

[173] Webby CJ, Wolf A, Gromak N, Dreger M, Kramer H, Kessler B (2009). Jmjd6 catalyses lysyl-hydroxylation of U2AF65, a protein associated with RNA splicing. Science.

[174] Unoki M, Masuda A, Dohmae N, Arita K, Yoshimatsu M, Iwai Y (2013). Lysyl 5-hydroxylation, a novel histone modification, by Jumonji domain containing 6 (JMJD6). J Biol Chem.

[175] Wang F, He L, Huangyang P, Liang J, Si W, Yan R (2014). JMJD6 promotes colon carcinogenesis through negative regulation of p53 by hydroxylation. PLoS Biol.

[176] Liu W, Ma Q, Wong K, Li W, Ohgi K, Zhang J (2013). Brd4 and JMJD6-associated anti-pause enhancers in regulation of transcriptional pause release. Cell.

[177] Chang B, Chen Y, Zhao Y, Bruick RK (2007). JMJD6 is a histone arginine demethylase. Science.

[178] Tibrewal N, Liu T, Li H, Birge RB (2007). Characterization of the biochemical and biophysical properties of the phosphatidylserine receptor (PS-R) gene product. Mol Cell Biochem.

[179] Wan J, Xu W, Zhan J, Ma J, Li X, Xie Y (2016). PCAF-mediated acetylation of transcriptional factor HOXB9 suppresses lung adenocarcinoma progression by targeting oncogenic protein JMJD6. Nucleic Acids Res.

[180] Lee YF, Miller LD, Chan XB, Black MA, Pang B, Ong CW (2012). JMJD6 is a driver of cellular proliferation and motility and a marker of poor prognosis in breast cancer. Breast Cancer Res.

[181] Prasad YD, Sonia S, Balvinder S, Charan CR (2013). Advanced glycation end products: A review. Sch Acad J Biosci.

[182] Ramasamy R, Yan SF, Schmidt AM (2011). Receptor for AGE (RAGE): signaling mechanisms in the pathogenesis of diabetes and its complications. Ann N Y Acad Sci.

[183] Kay AM, Rushing B, Simpson C, Stewart J (2017). AGE/RAGE Signaling in Diabetes-Mediated Vascular Calcification in Vascular Smooth Muscle Cells. FASEB J.

[184] P-c C, C-n H, C-c H, M-c Y, Guo Y-r (2010). Association of dietary AGEs with circulating AGEs, glycated LDL, IL-1α and MCP-1 levels in type 2 diabetic patients. Eur J Nutr.

[185] S-i Y, Nakamura N, Suematsu M, Kaseda K, Matsui T (2014). Advanced glycation end products: a molecular target for vascular complications in diabetes. Mol Med.

[186] Daffu G, Shen X, Senatus L, Thiagarajan D, Abedini A, del Pozo CH (2015). RAGE suppresses ABCG1-mediated macrophage cholesterol efflux in diabetes. Diabetes.

[187] Taguchi K, Yamagishi S-i, Yokoro M, Ito S, Kodama G, Kaida Y (2018). RAGE-aptamer attenuates deoxycorticosterone acetate/salt-induced renal injury in mice. Sci Rep.

[188] Hou B, Qiang G, Zhao Y, Yang X, Chen X, Yan Y (2017). Salvianolic acid a protects against diabetic nephropathy through ameliorating glomerular endothelial dysfunction via inhibiting AGE-RAGE signaling. Cell Physiol Biochem.

[189] Teismann P, Sathe K, Bierhaus A, Leng L, Martin HL, Bucala R (2012). Receptor for advanced glycation endproducts (RAGE) deficiency protects against MPTP toxicity. Neurobiol Aging.

[190] Suchal K, Malik S, Khan SI, Malhotra RK, Goyal SN, Bhatia J (2017). Protective effect of mangiferin on myocardial ischemia-reperfusion injury in streptozotocin-induced diabetic rats: role of AGE-RAGE/MAPK pathways. Sci Rep.

[191] Piperi C, Goumenos A, Adamopoulos C, Papavassiliou AG (2015). AGE/RAGE signalling regulation by miRNAs: associations with diabetic complications and therapeutic potential. Int J Biochem Cell Biol.

[192] He M, Kubo H, Morimoto K, Fujino N, Suzuki T, Takahasi T (2011). Receptor for advanced glycation end products binds to phosphatidylserine and assists in the clearance of apoptotic cells. EMBO Rep.

[193] Machahua C, Montes-Worboys A, Llatjós R, Escobar I, Planas L, Dorca J, et al. The ratio AGE/RAGE is increased in idiopathic pulmonary fibrosis. Eur Resp J. 2015;46:PA3811. 10.1183/13993003.congress-2015.PA3811.

[194] Yaser A-M, Huang Y, Zhou R-R, Hu G-S, Xiao M-F, Huang Z-B (2012). The role of receptor for advanced glycation end products (RAGE) in the proliferation of hepatocellular carcinoma. Int J Mol Sci.

[195] Radia A-M, Yaser A-M, Ma X, Zhang J, Yang C, Dong Q (2013). Specific siRNA targeting receptor for advanced glycation end products (RAGE) decreases proliferation in human breast cancer cell lines. Int J Mol Sci.

[196] Bao J-M, He M-Y, Liu Y-W, Lu Y-J, Hong Y-Q, Luo H-H (2015). AGE/RAGE/Akt pathway contributes to prostate cancer cell proliferation by promoting Rb phosphorylation and degradation. Am J Cancer Res.

[197] Ray R, Juranek JK, Rai V (2016). RAGE axis in neuroinflammation, neurodegeneration and its emerging role in the pathogenesis of amyotrophic lateral sclerosis. Neurosci Biobehav Rev.

[198] Phoenix DA, Harris F, Mura M, Dennison SR (2015). The increasing role of phosphatidylethanolamine as a lipid receptor in the action of host defence peptides. Prog Lipid Res.

[199] Emoto K, Toyama-Sorimachi N, Karasuyama H, Inoue K, Umeda M (1997). Exposure of phosphatidylethanolamine on the surface of apoptotic cells. Exp Cell Res.

[200] Yao Y, Huang C, Li Z-F, Wang A-Y, Liu L-Y, Zhao X-G (2009). Exogenous phosphatidylethanolamine induces apoptosis of human hepatoma HepG2 cells via the bcl-2/Bax pathway. World J Gastroenterol.

[201] Umeda M, Emoto K (1999). Membrane phospholipid dynamics during cytokinesis: regulation of actin filament assembly by redistribution of membrane surface phospholipid. Chem Phys Lipids.

[202] Carnec X, Meertens L, Dejarnac O, Perera-Lecoin M, Hafirassou ML, Kitaura J (2015). The phosphatidylserine and phosphatidylethanolamine receptor CD300a binds dengue virus and enhances infection. J Virol.

[203] Stafford JH, Thorpe PE (2011). Increased exposure of phosphatidylethanolamine on the surface of tumor vascular endothelium. Neoplasia.

[204] Barnett Foster D, Abul-Milh M, Huesca M, Lingwood CA (2000). Enterohemorrhagic Escherichia coli induces apoptosis which augments bacterial binding and phosphatidylethanolamine exposure on the plasma membrane outer leaflet. Infect Immun.

[205] Richard AS, Zhang A, Park S-J, Farzan M, Zong M, Choe H (2015). Virion-associated phosphatidylethanolamine promotes TIM1-mediated infection by Ebola, dengue, and West Nile viruses. Proc Natl Acad Sci.

[206] Mayor J, Torriani G, Zimmer G, Rothenberger S, Engler O. T-cell immunoglobulin and mucin (TIM) contributes to Hantaan virus entry into human airway epithelial cells. bioRxiv. 2019:872317.

[207] Sciacca MFM, Brender JR, Lee D-K, Ramamoorthy A (2012). Phosphatidylethanolamine enhances amyloid fiber-dependent membrane fragmentation. Biochemistry.

[208] Tavoosi N, Davis-Harrison RL, Pogorelov TV, Ohkubo YZ, Arcario MJ, Clay MC (2011). Molecular determinants of phospholipid synergy in blood clotting. J Biol Chem.

[209] Bazzi MD, Nelsestuen GL (1993). Protein kinase C and annexins: unusual calcium response elements in the cell. Cell Signal.

